# Cardiac Fibroblasts Promote Ferroptosis in Atrial Fibrillation by Secreting Exo-miR-23a-3p Targeting SLC7A11

**DOI:** 10.1155/2022/3961495

**Published:** 2022-05-29

**Authors:** Dishiwen Liu, Mei Yang, Yajun Yao, Shanqing He, Youcheng Wang, Zhen Cao, Huiyu Chen, Yuntao Fu, Huafen Liu, Qingyan Zhao

**Affiliations:** ^1^Department of Cardiology, Renmin Hospital of Wuhan University, Wuhan 430060, China; ^2^Cardiovascular Research Institute, Wuhan University, Wuhan 430060, China; ^3^Hubei Key Laboratory of Cardiology, Wuhan 430060, China

## Abstract

The exact mechanism of atrial fibrillation (AF) has been not well elucidated. Ferroptosis is an iron-dependent cell death due to excessive accumulation of peroxidized polyunsaturated fatty acids. However, the molecular mechanism underlying AF and ferroptosis has never been reported. Here, we established the rapid pacing model in vivo and vitro to investigate the relationship between AF and ferroptosis. In canine model of rapid atrial pacing, the content of malondialdehyde and total ions in the atrial tissue of the Pacing group was significantly increased and the exosome inhibitor GW4869 reduced ferroptosis, fibrosis, and inflammation and improved histological and electrophysiological remodeling. In rapid pacing h9c2 cells, the expression of antioxidative stress genes associated with ferroptosis presented sequential changes and proteins involved in ferroptosis such as FTH1, SLC7A11, and GPX4 were gradually depleted. Furthermore, pacing cardiac fibroblast-derived exosomes (CF-exos) exacerbated ferroptosis in h9c2 cells and pretreated pacing-CF-exos with GW4869 alleviated injury to h9c2 cells. In mechanism, our results demonstrated that pacing-CF-exos highly expressed miR-23a-3p by informatics analysis and experimental verification. Inhibitor-miR-23a-3p protected h9c2 cells from ferroptosis accompanying with upregulation of SLC7A11. In addition, SLC7A11 was shown to be the target gene of miR-23a-3p. In conclusion, our results suggest that CF-exos-miR-23a-3p may promote ferroptosis. The development of AF in a persistent direction could be prevented by intervening with exosomal miRNAs to reduce oxidative stress injury and ferroptosis.

## 1. Background

As atrial fibrillation (AF) incidence has increased in recent decades, AF and its complications, such as heart failure and stroke, pose a serious public health threat [1]. Although the most effective physical approach is radiofrequency ablation, no therapies have been developed for the targeted treatment of its pathophysiological mechanism. Current research suggests that renin-angiotensin-aldosterone system (RAAS) activation, inflammation, oxidative stress, apoptosis, and autonomic imbalance are all involved in the maintenance of AF [2, 3].

In AF intricate pathophysiological network, oxidative stress and fibrosis are the central mechanisms and these mechanisms could interact [4]. Reactive oxygen species (ROS) activate a wide variety of fibrogenic signaling and transcription factors, which stimulates cardiac fibroblast proliferation and matrix remodeling. Besides, excessive ROS also leads to ion remodeling and apoptosis [5]. Recent studies have shown that hypoxia induces HL-1 cardiomyocytes to secrete hypoxia-inducible factors through the JNK/ROS signaling pathway, which expedites fibrosis and provides a matrix for the occurrence of AF [6]. In addition, Angiotensin (Ang) II promotes the susceptibility of AF by inducing *α*1C subunit of L-type calcium channel promoter activity through a PKC/NADPH oxidase/ROS pathway [7]. The homeostasis of Ca^2+^ in cells is critical for the maintenance of mitochondrial function. Ca^2+^ handling abnormity causes profound decrease of mitochondrial membrane potential (MMP) and adenosine triphosphate, and the increase of ROS derived from mitochondria, leading to cell death [5]. The loss of atrial cardiomyocytes caused by electrophysiological disorders forms a vicious circle that drives AF progress in a sustained direction. Undeniable, the major protective mechanism against oxidative stress damage in cells is to restore redox homeostasis by increasing the expression of antioxidant-related genes and proteins such as FTH1, GPX4, SLC7A11, and antioxidant enzymes [8–10].

Ferroptosis is an iron-dependent cell death that is different from apoptosis and necrosis due to excessive accumulation of peroxidized polyunsaturated fatty acids, which are principally oxidized polyunsaturated fatty acids by ROS through the Fenton reaction [11]. Current evidence verified that ferroptosis occurs in a wide variety of cells and prevails in myocardial tissue of pathological condition [12]. In the mouse model of ischemia/reperfusion, iron chelator deferoxamine and ferrostatin (Fer-1) reduced myocardial infarction size and preserved heart function [13]. Coincidentally, cardiomyocytes who experienced ferroptosis after ischemia/reperfusion in heart transplantation stimulated the recruitment of neutrophils through the TLR4/TRIF/IFN signaling pathways and caused inflammation in regional myocardial tissues [14]. Tadokoro et al. reported doxorubicin downregulated GPX4 in mitochondria, leading to mitochondria-dependent ferroptosis [15]. Similarly, electrophysiological disorders also cause mitochondrial malfunction and the accumulation of ROS. Based on those evidence, we hypothesized that ferroptosis occurs in AF.

Exosomes, which can be secreted by almost all cells, are extracellular vesicles with a diameter of 30-150 nm. Donor cells exchange information with recipient cells through exosomes encapsulating miRNA, mRNA, DNA, and bioactive molecules. Interestingly, cells also wrap metabolites in exosomes and excrete extracellular to resist external stimuli. For instance, prominin 2 promotes ferritin-containing exosomes to transport iron out of mammary epithelial cells and breast carcinoma cells, inhibiting ferroptosis [16]. Nonetheless, pernicious exosomes may have detrimental effect on those vulnerable recipient cells. Studies have reported that exosomes from Ang II-treated cardiac fibroblasts (CFs) contained hypertrophic molecules that induced the release of renin and Ang II in cardiomyocytes [17]. In addition, recent studies found that exosomes isolated from the plasma of patients with AF significantly suppressed human umbilical vein endothelial cell viability and migration and enhanced cell apoptosis [18]. GW4869, which is a specific, noncompetitive inhibitor of neutral sphingomyelinase, can reverse this process [19]. Meanwhile, previous studies found that the inhibitor of sphingomyelinase could alleviate the fibrosis [20, 21]. In our recent study, we also found that blockade of exosome release suppressed AF and atrial fibrosis [22].

However, to the best of our knowledge, whether AF can trigger ferroptosis and the effects of ferroptosis on AF vulnerability have not been evaluated. The purpose of this study was to test the hypothesis that exosomes regulated ferroptosis is the key to the maintenance of AF.

## 2. Materials and Methods

### 2.1. Microarray Data

The array data of GSE2240, GSE14975, GSE31821, GSE41177, GSE79768, GSE115574, GSE128188, GSE138252, and GSE143924 were downloaded from the Gene Expression Omnibus (GEO) database. A total of 128 normal atrial tissue samples and 139 AF atrial tissue samples were included. The merged, DMwR, lattice, and grid packages in the R statistical software were used to eliminate 50% of the genes lacking in the raw data. Background correction, normalization, and a calculating expression were included in the process of preprocessing. Finally, a total of 20730 gene expression values were obtained. For miRNA expression, the array data of GSE28954, GSE68475, and GSE70887 were also downloaded from the GEO database. 33 normal atrial tissue samples and 30 AF atrial tissue samples were included. By using similar methods above to process the raw data, a total of 383 miRNA expression values were obtained. The limma package was used to analyze the differentially expressed genes (DEGs) analysis in AF samples compared with control samples. In the analysis process, the *P*-values of the DEGs were calculated using eBayes tests in the limma package. |log2FC| ≥ 1 and adj *P* < 0.05 were used as cut-off criteria. Kyoto Encyclopedia of Genes and Genomes (KEGG) pathway enrichment analysis was performed.

### 2.2. Animal Model Preparation

This study was approved by the animal research committee of our institutional review board and is in line with NIH guidelines for the care and use of laboratory animals. Eighteen beagles, randomly divided into three groups, both sexes and an average age of 1 year, weighing 7.5 ± 1.5 kg, were used for the study as follows: Sham group (*n*=6), Pacing group (*n*=6), and GW4869+Pacing group (*n*=6). Each beagle canine was given an intramuscular injection of 25 mg/kg ketamine sulfate before being premedicated with pentobarbital sodium (30 mg/kg, intravenous injection) and ventilated with room air by a respirator (MAO01746, Harvard Apparatus Holliston, United States). Venous access was established to supply saline (50-100 mL/h) or pentobarbital sodium (2.5 mg/kg/h). Standard body surface ECG leads (I, II, and III) were monitored continuously throughout the procedure. Under fluoroscopy, an atrial endocardial pacing electrode (St Jude Medical, United States) was delivered to the right atrial appendage via the right external jugular vein and connected to a high-rate cardiac pacemaker (450 bpm, Harbin University, China), which was implanted in a subcutaneous pocket of the neck. The incision was covered with sterile gauze, and 4 million units of penicillin were injected intramuscularly for 3 consecutive days after the operation. After 3 days of recovery, the GW4869+Pacing group was given an intravenous injection of GW4869 (0.3 mg/kg/d, MCE, United States). The Pacing group and GW4869+Pacing group were paced at 450 bpm for 7 days.

### 2.3. Electrophysiological Measurements

All canines were anesthetized again after 7 days and bilateral thoracotomy was performed. Multielectrode catheters (Biosense-Webster, Diamond Bar, United States) were secured to discrete part of the atrium. All recordings were documented on a computerized electrophysiology system (Lead 7000, Jinjiang Inc., China). The atrial effective refractory period (ERP) was measured by delivering a train of eight atrial paced beats S1 at a cycle length of 250 ms, followed by an extra stimulus (S2) introduced at coupling intervals. The S1-S2 intervals were decreased from 180 ms to refractoriness initially by decrements of 10 ms. As the S1-S2 intervals approached the ERP, decrements were reduced to 2 ms. The dispersion of the ERP (dERP) was calculated as the maximum ERP minus the minimum ERP at all recording sites. The inducibility and duration of AF were assessed using programmed S1S1 stimulation (a 5 s burst at cycle length of 120, 100, 75, and 60 ms, three times at every frequency). AF was defined as an irregular atrial rate of >500 bpm, lasting for >5 s [23]. AF inducibility and AF duration were determined by the number of episodes and the maximum duration induced by all bursts of every canine, respectively.

### 2.4. Histological Analysis

Canine atria tissue was fixed with 4% formaldehyde overnight. Then, it was embedded in paraffin and cut into 5 *μ*m sections. For Prussian blue staining, atrial sections were deparaffinized at 60°C for 1 h and hydrated in distilled water. Equal volumes of potassium ferrocyanide solution and hydrochloric acid solution were mixed to make a working iron stain solution. The sections were then incubated with the working solution for 3 min. For hematoxylin & eosin (H&E) staining, the sections were stained with hematoxylin for 10 min and then stained with aniline blue solution for 5 min, followed by staining with 1% acetic acid solution for 2 min. To detect FTH1 or SLC7A11, 3% H_2_O_2_ and 5% goat serum were used. Subsequently, the sections were incubated with FTH1 antibodies (Bios, bs-8679r; 1 : 200) and SLC7A11 (Proteintech, 26864-1-ap; 1 : 200) at 4°C overnight. Finally, the sections were incubated with a horseradish peroxidase-conjugated goat antirabbit IgG secondary antibody (Aspen, as1110; 1 : 200) at 37°C for 50 min and DAPI at room temperature for 5 min.

### 2.5. ROS and JC-1

MMP and ROS were evaluated using the JC-1 Assay Kit (MCE, United States) and ROS Assay Kit (Biorbyt, China), respectively. Cells in 6-well plates were harvested or resuspended in 1 mL DMEM/F12. 1 mL sample of the cell suspension was mixed with 10 *μ*L JC-1 or 5 *μ*L DCFH-DA. The mixture was incubated for 15 min or 20 min at 37°C in the dark and then washed once with ice-cold 1× binding buffer. Subsequently, the cells were analyzed by a FACSCalibur flow cytometer (BD United States).

### 2.6. Malondialdehyde (MDA) and Total Iron in Atrial Tissue and Cells

The levels of MDA or total iron in atrial tissue and cells were detected by a lipid peroxidation MDA assay kit (Biorbyt, China) and iron detection kit (Leagene, China), respectively. Samples were read at 532 nm or 562 nm using colorimetric determination (Tecan, Switzerland) according to the manufacturer's instructions.

### 2.7. Western Blotting (WB)

Total protein was extracted from the atria tissue and cells by RIPA lysis buffer (Servicebio, g2002), and the protein concentration was determined by a BCA Protein Assay Kit (Aspen, as1086) according to the manufacturer's instruction. After mixing with loading buffer, protein samples were denatured in a boiling water bath for 10 minutes. Protein samples were separated on SDS-PAGE gels (10%), then transferred to PVDF membranes (0.45 *μ*m, Millipore). QuickBlock (Epizym, ps108) was used to block for 10-20 minutes. Subsequently, the membranes were incubated with primary antibodies against GAPDH (Abcam, ab181602; 1 : 10000), Cav1.2 (Alomone, acc-003; 1 : 500), KCa3.1 (Bioss, bs-6675r; 1 : 500), CD63 (Biorbyt, orb11597; 1 : 1000), CD81 (Abcam, ab109201; 1 : 1000), TSG101 (Sigma, av38773; 1 : 500), FTH1 (Abcam, ab65080; 1 : 1000), GPX4 (Abcam, ab125066; 1 : 1000), and SLC7A11 (Biorbyt, orb325112; 1 : 500) overnight at 4°C. Then, the membranes were incubated with the secondary horseradish peroxidase-conjugated antibody (Proteintech, pr30012; 1 : 3000) at room temperature for 1 hour. GAPDH was used as a control to normalize the signal intensities. The AlphaEase FC software system was used to analyze the optical density value.

### 2.8. Quantitative Real-Time PCR

Total RNA was extracted from the atrial tissue or cell using TRIzol® reagent (Takara, Japan). Isolated RNA (2 *μ*g) was converted into complementary DNA using an RT First Strand cDNA Synthesis Kit (Servicebio, China). The mRNA was reverse transcribed using Oligo (dT) primers. Since primers were designed by the stem-loop methods, each miRNA reverse transcription needs to add the corresponding reverse transcription primer for reverse transcription (Table 1). The cDNA templates were amplified by qRT-PCR system (Applied Biosystem, United States) using SYBR Green PCR Mix (Servicebio, China) with the corresponding primers (Table 1). The 2^-*ΔΔ*Ct^ comparative quantification method was used to analyze the semilog amplification curves, and the expression of gene and miRNA were normalized to GAPDH and U6, respectively.

### 2.9. Isolation of CFs and Transfection

Ventricular cells were isolated from 3-day-old Sprague-Dawley neonatal rat as previously described [24]. Ventricular cells were cultured in DMEM/F12 supplemented with 15% fetal bovine serum (BI, Israel) and 1% penicillin-streptomycin for 1.5 hours. CFs and cardiomyocytes were separated by postdifferential adhesion. hsa-miR-23a-3p mimics (5′-AUCACAUUGCCAGGGAUUUCC-3′), hsa-miR-23a-3p inhibitor (5′-GGAAAUCCCUGGCAAUGUGAU-3′), and their corresponding negative controls (NC mimics; 5′-UCACAACCUCCUAGAAAGAGUAGA-3′; NC inhibitor; 5′-UCUACUCUUUCUAGGAGGUUGUGA-3′) were synthesized by General Biol, China. Mimics/inhibitor-miR-23a-3p were transfected using Lipofectamine 6000 (Biorbyt, China). Cells were harvested for further experiments after 24 h.

### 2.10. Preparation of AF Cell Model

CFs or h9c2 cells were processed after their growth reached approximately 60%-80%. A carbon electrode with a diameter of 2 mm was sterilized at high temperature. Subsequently, electric soldering iron was used to punch holes on both sides of the petri dish, and the carbon electrode was placed in the petri dish to contact the culture medium. After the carbon electrode connected to the stimulation system (Master 8, Israel), it was stimulated with an electric field of 1.0 v/cm and a frequency of 10 Hz, and the cells were harvested after 12-72 h.

### 2.11. Exosome Isolation

Exosomes were isolated by gradual differential centrifugation. Large cells, debris, and other vesicles were removed by centrifugation at 300 g, 3000 g, and 10000 g, respectively. Subsequently, the supernatant was centrifuged at 120000 g for 90 min (Beckman Coulter, Optima XPN, United States). Finally, the obtained exosomes were resuspended in 100 *μ*L PBS.

### 2.12. Luciferase Reporter Assay

Luciferase reporter constructs were generated by inserting the human species WT SLC7A11 3′UTR or Mut ALOXE3 3′UTR into the pmirGLO vector (Addgene, e1330, United States). 293T cells were transfected with the indicated luciferase vectors and miRNAs using Lipofectamine 2000 (Thermo, United States). After 48 hours transfection, Firefly/Renilla dual-luciferase activity was determined by dual-luciferase reporter assay (Promega, United States).

### 2.13. Statistical Analysis

Statistical analyses were performed using SPSS 25.0 software (IBM, United States) or GraphPad Prism 8.0 (GraphPad Software, Inc., United States). The data are presented as the mean ± SD (standard deviation). Two-tailed Student's *t*-test or one-way ANOVA was implemented to determine differences. A *P* < 0.05 was considered to indicate a statistically significant difference.

## 3. Results

### 3.1. Exosomes Involved in AF

After quality detection of microarray raw data, a total of 34 DEGs were obtained in the merged dataset. Among these DEGs, 6 genes were upregulated and 28 genes were downregulated (Figures 1(a) and 1(b)). The DEGs were involved in extracellular exosome in cellular component analysis. KEGG pathway analysis found that the DEGs were mainly enriched in the sphingolipid signaling pathway (Figures 1(c) and 1(d)). In the process of intravenous systemic administration of GW4869, although we did not conduct detailed tests on the blood biochemistry of canines, we did not find discernible adverse effects, including incontinence, diarrhea, decreased appetite, increased secretion, and abnormal behavior. We did not observe spontaneous AF in canines after 7 days of rapid atrial pacing.

### 3.2. GW4869 Inhibited the Electrical Remodeling and AF Vulnerability in Canines with Rapid Atrial Pacing

In order to survey the efficacy of GW4869 on the in vivo electrophysiology of rapid atrial pacing in canines, we measured the ERP of different parts of the atrium. Overall, the ERP of the Pacing group was significantly shorter than that of the Sham group. After using GW4869, the ERPs of the right superior pulmonary vein and left inferior pulmonary vein were higher than that of the Pacing group. Compared with Pacing group, although the ERP of other parts of the atrial tissue tended to increase in the GW4869+Pacing group, there was no significant difference (Figure 2(b)). In addition, the number of inductions and the duration of AF were highest in the Pacing group, while GW4869 was lower than that of the Pacing group (Figures 2(a), 2(c), and 2(d)). The ion channel, voltage-gated L-type calcium channel (Cav1.2), was significantly reduced in the Pacing group, while the expression of potassium intermediate conductance calcium-activated channel (KCa3.1) was increased, and GW4869 reversed these effects (Figures 2(e) and 2(f)).

### 3.3. GW4869 Reduced Exosome Secretion, Fibrosis, Inflammation, and Ferroptosis in Canines with Rapid Atrial Pacing

Previous studies found that macrophages treated with lipopolysaccharide increased the release of exosomes and proinflammatory factors such as TNF-*α*, IL-1*β*, and IL-6, while GW4869 can reverse this process [25]. Similarly, our result found that the exosome markers CD63, CD81, and TSG101 in the Pacing group were significantly higher than those in the Sham group. Not surprisingly, the use of GW4869 significantly decreased these markers (Figures 3(a) and 3(b)). Hence, our results verified that the secretion of exosomes increased under the pathological condition of rapid pacing. H&E staining demonstrated apparent inflammatory cells infiltration in the Pacing group, and GW4869 mitigated inflammation (Figure 3(d)). Masson staining indicated prominent fibrosis and collagen deposition in the Pacing group, while GW4869 also alleviated this process (Figures 3(d) and 3(f)).

Experimental evidence supported that acute myocardial infarction and doxorubicin-induced cardiomyopathy lead to ferroptosis in cardiomyocytes [15, 26], but there are currently no research data to prove that ferroptosis also occurs in AF. To verify whether ferroptosis occurred in AF, we examined relevant genes related to ferroptosis at the mRNA and protein levels. In the Pacing group, GPX4 and SLC7A11 were significantly decreased in transcription and translation, while GW4869 prevented the degradation of GPX4 and SLC7A11 (Figures 3(a), 3(c), and 3(h)). Meanwhile, immunohistochemical results also showed that SLC7A11 was significantly decreased in the Pacing group (Figure 3(d)). Lipid peroxidation increases the proportion of lipid alkoxies such as MDA. Likewise, there was an increase in MDA in the Pacing group, and it was reduced by GW4869 (Figure 2(h)). As ferritin heavy chain 1 (FTH1) is an important iron storage protein in cells, it indicates the occurrence of ferroptosis [27]. Our results demonstrated that rapid pacing led to the degradation of FTH1 at the transcriptional and translational levels, which was also confirmed by immunofluorescence, while GW4869 alleviated the degradation of FTH1 (Figures 3(a), 3(c), 3(e), and 3(g)). In addition, rapid pacing increased total iron in the atrial tissues, and GW4869 reduced this effect (Figure 2(g)). Prussian blue-stained positive cells were significantly increased in the Pacing group, but GW4869 reduced such positive cells, indicating that GW4869 partially inhibits ferroptosis (Figure 3(d)).

### 3.4. Fer-1 Alleviates Cardiomyocytes Ferroptosis in Rapid Pacing Cell Model

To explore which cells experienced ferroptosis in the myocardial tissue, we used h9c2 cells and CFs for rapid pacing. h9c2 cells have a significant effect on rapid pacing. Although we did not observe apparent pulsation during electrical stimulation, we observed difficulty in adherence of cells, and the cells were suspended as the increased voltage and the frequency. This may be related to the reduction of cell surface caused by electrical stimulation [28].

In our rapid pacing h9c2 cells model, we found that the transcription level of genes involved in ferroptosis changed dramatically over time. FTH1, GPX4, and SLC7A11 increased in the early stage of pacing, where FTH1 reaches its peak at approximately 24 hours and then gradually decreases (Figure 4(a)). The peaks of GPX4 and SLC7A11 appeared earlier and then showed a consistent downward trend (Figures 4(b) and 4(c)). Interestingly, FTL decreased from the beginning of pacing, and then the expression did not change much over time (Figure 4(d)). We chose 48 hours as the time point to observe the changes in FTH1 at the protein level. The protein expression of FTH1 was consistent with the mRNA expression, and FTH1 gradually returned to baseline (Figures 4(e) and 4(f)), which was also confirmed by immunofluorescence (Figures 4(i) and 4(k)), but total iron was significantly increased in the Pacing group (Figure 4(o)). However, the protein expression of GPX4 and SLC7A11 was significantly reduced and could be improved by Fer-1 (Figures 4(e) and 4(f)). Interestingly, when the continuous pacing reached 72 hours, the antioxidant genes involved in ferroptosis were exhausted at the transcription and translation levels. The expression of FTH1 decreased significantly in the Pacing group, which is consistent with the results of our vivo experiments, and Fer-1 alleviated the degradation of FTH1, GPX4, and SLC7A11 (Figures 4(g) and 4(h)). Hence, cardiomyocytes may initially resist to rapid pacing-induced ferroptosis. If hazards are not eliminated, those compensatory mechanisms will be gradually exhausted.

In parallel experiments, we found that the MMP in the Pacing group was significantly reduced, but this was alleviated by Fer-1 (Figures 4(m) and 4(n)). As indicators of oxidative stress, our results demonstrated that the levels of ROS and MDA related to lipid peroxidation in the Pacing group were significantly increased, and this process could also be inhibited by Fer-1 (Figures 4(j), 4(l), and 4(p)). In addition to reducing oxidative stress damage, Fer-1 also improved ion channel remodeling. Compared with the Pacing group, the expression of Cav1.2 increased and KCa3.1 decreased in the Fer-1+Pacing group (Figures 4(q) and 4(r)).

### 3.5. Exosomes Secreted by Pacing CFs Promote Ferroptosis in h9c2 Cells

CFs are inherently nonexcitable cells, but it makes pathophysiological changes to rapid pacing. After 48 hours of rapid pacing, we observed an increase in CFs branching with a tendency to differentiate into myofibroblasts [29]. To explore the specific mechanism of GW4869 inhibiting ferroptosis, we isolated cardiac fibroblast-derived exosomes (CF-exos) from equal amounts of supernatant at the same cell density to coincubate with h9c2 cells. The morphology and particle size were observed by transmission electron microscope and nanoparticle tracking analysis, respectively. Transmission electron microscope showed that isolated CF-exos were extracellular vesicles with a diameter of 35-143 nm (Figure 5(a)). The size of the vesicles ranged between 50 and 300 nm, most of which were 100-150 nm in diameter (Figure 5(b)). Consequently, the tested sample obtained by ultracentrifugation conformed to the structure and particle size of exosomes.

Coincubating the collected CF-exos with h9c2 cells, we found that the exosomes can be engulfed by h9c2 cells and enter the cytoplasm (Figure 5(c)). Strikingly, in the coincubation experiment, normal CF-exos may even nourish cardiomyocytes. At the protein level, FTH1 did not change significantly, but both GPX4 and SLC7A11 decreased in the pacing-CF-exo group, and Fer-1 could partly restore this decrease (Figures 5(d) and 5(e)). The increase of MDA and intracellular total iron was most obvious in the pacing-CF-exos group, and Fer-1 antagonized this change. In addition, the MDA and intracellular total iron of the GW4869-pacing-CF-exos group were lower than those of the pacing-exos group (Figures 5(f) and 5(g)). At the level of oxidative stress, ROS increased in the pacing-exo group, while Fer-1 protected h9c2 cells from the vicious effects of pacing-CF-exos. Meanwhile, pacing-CF-exos treated with GW4869 reduced the production of ROS in h9c2 cells (Figures 5(j) and 5(k)). Moreover, the proportion of early apoptosis was the highest in the pacing-CF-exos group, and both GW4869 and Fer-1 significantly increased the MMP (Figures 5(h) and 5(i)). As expected, pacing-CF-exos had a pernicious effect on cardiomyocytes, while GW4869 partially alleviated this side effect. GW4869 may interfere with the communication between CFs and cardiomyocytes by reducing the quantity of exosomes.

### 3.6. miR-23a-3p Increased in Human Atrial Tissue, Canine Atrial Tissue, and CF-Exos

Based on the current research evidence, we believe that miRNA in exosomes may play a vital role in signal transduction between cells. To further explore the specific substances in exosomes that caused ferroptosis, we first screened miRNAs by bioinformatics. A total of 62 differentially expressed miRNAs in human atrial tissue were obtained in the merged dataset. Among these differentially expressed miRNAs, 53 miRNAs were upregulated and 9 miRNAs were downregulated (Figures 6(a) and 6(b)).

After screened out differentially expressed miRNAs, we investigated the top 8 miRNAs with significant differences. Unexpectedly, miRNA expression in canine atrial tissue verified by RT-PCR was not completely consistent with bioinformatic analysis. cfa-miR-21/23 was significantly increased after pacing, and GW4869 inhibited its expression. Nevertheless, cfa-let-7 and cfa-miR-15 decreased in Pacing group, while GW4869 increased its expression. The expression of cfa-miR-30 decreased in Pacing group, while GW4869 seemed to have no effect on it. cfa-miR-199 tended to increase in Pacing group, while there was no significant difference, but GW4869 significantly increased its expression (Figure 6(c)). These results may be attributed to the short time of rapid atrial pacing. To verify the differential expression of miRNA between cells, we paced CFs and h9c2 cells and treated with GW4869. Our results uncovered that miRNA expression of h9c2 cells did not change significantly after pacing (Figure 6(d)). However, rno-miR-23a-3p and rno-miR-199a increased after pacing in CFs, and GW4869 reduced its levels. Interestingly, the use of GW4869 increased rno-miR-15 in CFs (Figure 6(e)). To substantiate whether rno-miR-23a-3p is encapsulated in CF-exos, we performed RT-PCR verification in CF-exos. We found that rno-miR-23a-3p was also significantly elevated in pacing-CF-exos, and GW4869 reversed this effect (Figure 6(f)). Thus, we confirmed that the exosome inhibitor GW4869 not only changes the quantity of exosomes but also its quality.

### 3.7. Rno-miR-23a-3p Promotes Ferroptosis in h9c2 Cells

Gain and loss of function experiments were performed to explore the effect of rno-miR-23a-3p on cardiomyocytes. After 48 hours of transfected mimics or inhibitor-23a-3p into h9c2 cells, respectively, we verified the transfection efficiency by RT-PCR. Interestingly, inhibitor-miR-23a did not significantly alter the level of rno-miR-23a-3p (Figure 7(a)). Inhibitor-miR-23a-3p may mainly manipulate the biological function of rno-miR-23a-3p. Moreover, we detected the baseline level of SLC7A11 mRNA expression after transfection. Our results revealed that mimics-miR-23a-3p significantly reduced the expression of SLC7A11 mRNA, while inhibitor-miR-23a-3p had the opposite effect (Figure 7(b)). To further explore whether excessive rno-miR-23a-3p could induce ferroptosis on h9c2 cells, we tested MDA and intracellular total iron. The results showed that both of them were significantly increased in the mimics group, and Fer-1 exhibited a protective effect (Figures 7(c) and 7(d)). The JC-1 results confirmed that mimics-miR-23a-3p reduced the MMP of h9c2 cells, and Fer-1 reversed this adverse effect (Figures 7(e) and 7(f)). Furthermore, when suppressing the expression of SLC7A11 mRNA, mimics-miR-23a-3p synchronously reduced FTH1 and GPX4 at the protein level, and Fer-1 ameliorated the degradation of these protective factors (Figures 7(g) and 7(h)). In contrast, inhibitor-miR-23a-3p increased the expression of antioxidant proteins such as FTH1, GPX4, and SLC7A11 (Figures 8(a) and 8(b)). In Pacing group, ROS, intracellular total iron, and MDA were significantly elevated, while inhibitor-miR-23a-3p antagonized these changes (Figures 8(c), 8(d), 8(g), and 8(h)). In addition, the use of inhibitor-miR-23a-3p increased MMP in Pacing group (Figures 8(e) and 8(f)). Using the online prediction website starBase, we found that hsa-miR-23a-3p may target multiple sites of the SLC7A11 mRNA (Figure 8(i)). Mimics-miR-23a-3p significantly decreased the activity of luciferase harboring the wild-type SLC7A11 3′UTR vector. However, it had no effect on the luciferase activity of the vector with the mutant SLC7A11 3′UTR (Figure 8(j)). These results suggested that hsa-miR-23a-3p could directly target the 3′UTR of SLC7A11. Overall, inhibitor-miR-23a-3p could promote a certain resistance to ferroptosis in cardiomyocytes.

## 4. Discussion

This study explored the function of the exosome inhibitor GW4869 in vivo and in vitro to verify the relationship between AF, exosomes, and ferroptosis. We provide evidence for the following: (1) GW4869 suppresses atrial electrical and structural remodeling in a pacing-induced AF model by inhibiting fibrosis, inflammation, and ferroptosis; (2) miR-23a-3p encapsulated by CFs exosomes promoting the ferroptosis of cardiomyocytes by inhibiting the transcription of SLC7A11 mRNA and depleting the Xc^−^ transport system.

Fibrosis plays a crucial role in AF structure and electrical remodeling, and it is the final outcome of various mechanisms, which has been confirmed in numerous studies. For instance, activation of TGF-*β*/SMAD and Ang II signaling pathways promote fibrosis by generating ROS. Proinflammatory factors such as IL-1, 6, and chemokines activate fibroblasts, leading to myofibroblast proliferation and the deposition of extracellular matrix. Atrial fibrosis increases the anisotropy of conduction and shortens action potential duration (APD), making it easier to maintain AF. The interaction between oxidative stress and fibrosis impels the progression of AF towards persistence. Nevertheless, blocking communication between cells via exosomes may abrogate fibrosis. Qin et al. found that silica-exposed macrophage-derived exosomes promoted fibroblast differentiation, proliferation, and migration. Their vivo study demonstrated that pre-treatment with GW4869 decreased lung fibrosis and the expression of TNF-*α*, IL-1*β*, and IL-6 in silicosis model [20]. In addition, it has been reported macrophage exosomes transferred Ang IIR to lung fibroblasts mediating bleomycin-induced pulmonary fibrosis, which is damped by GW4869 [21]. Our previous study also confirmed that GW4869 reduced the induction of AF by inhibiting atrial fibrosis [22]. All these results suggest that in pathological condition, exosome secretion increased for intercellular communication leads to disease progression. There may be benefits to blocking this interaction.

Oxidative stress increases risk for cardiomyocytes injury/death, inflammation, and fibrosis. In AF canine model, atrial rapid pacing for two weeks increased the oxidative stress and inflammation indicator [30]. More evidence suggests that AF induces calcium accumulation in mitochondria leading to increased oxidative stress [31, 32]. Our in vivo and in vitro experiments also yielded analogous results. Rapid pacing increases the oxidative stress products and significantly depletes the antioxidant system, and the antioxidant Fer-1 protects cardiomyocytes from oxidative stress injury.

Oxidative stress-driven plasma membrane peroxidation is associated with ferroptosis characterized by iron overload. Ferroptosis apparently occurs more commonly in myocardial infarction and heart failure. For example, hypoxia/reoxygenation regulates cardiomyocytes ferroptosis through Nrf2/HO-1 signaling pathway [33]. Ma et al. found USP22 protected against myocardial ischemia/reperfusion injury via the SIRT1-p53/SLC7A11 dependent inhibition of ferroptosis [34]. Recent studies found that FTH1 knockout mice spontaneously developed heart failure and induced cardiomyocytes ferroptosis through SLC7A11, confirming that the FTH1 is crucial in ferroptosis [27]. In addition, downregulation of GPX4 also promotes ferroptosis in cardiomyocytes [26, 35]. Nevertheless, it has never been reported whether disturbances in electrophysiology lead to ferroptosis. Our study substantiates that ferroptosis occurs in AF. Correspondingly, the expression of antioxidant genes was significantly reduced both in vivo and in vitro after rapid pacing. Besides, our result demonstrated that the alteration of FTH1 has a hysteresis, and GPX4 and SLC7A11 are more susceptible to oxidative stress. With prolonged unfavorable stimulation, this protective mechanism is gradually depleted.

In terms of specific mechanisms, our findings confirm that exosomes are involved in the occurrence of ferroptosis in AF. At present, studies have found that stem cell-derived exosomes enhanced the repair of cardiomyocytes after myocardial infarction. These exosomes enhanced angiogenesis and cardiomyocytes survival, and reduced fibrosis [36, 37]. Nevertheless, exosomes from AF patients' epicardial fat harbor large amounts of proinflammatory and profibrotic cytokines, and profibrotic miRNA, which shortened the APD of cardiomyocytes [38]. Li et al. demonstrated that CF-exos increased the susceptibility of AF by downregulation of Cav1.2 expression in cardiomyocytes [39]. CFs, which are the main initiating factors of fibrosis, occupy 60% of the cellular components of myocardial tissue, and have adverse effects on cardiomyocytes under pathological conditions. Our research verified that interfering with the collaboration between cardiomyocytes and CFs reduced inflammation, fibrosis, and ferroptosis in rapid pacing AF model. Furthermore, pacing-CF-exos increased the accumulation of ROS, lipid peroxidation, and iron content and reduced the MMP in cardiomyocytes.

System Xc^−^, which consists of the light chain subunit SLC7A11 and heavy chain subunit SLC3A2, is a cystine/glutamate antiporter on the cell surface and mediates the uptake of extracellular cystine. More importantly, SLC7A11 is specific for System Xc^−^, while SLC3A2 is the chaperone protein [40]. SLC7A11 regulates the uptake of cysteine and is considered the rate-limiting step in glutathione biosynthesis. Interestingly, as predicted by starBase and TargetScan, we found that nearly 75% of the upregulated miRNAs we identified by bioinformatics analysis could target SLC7A11. Studies suggested that mmu-miR-23 inhibited tumor proliferation and invasion. To a certain extent, it serves as a tumor suppressor gene [41]. The role of dre-miR-23a in the formation of embryonic myocardium has been well studied. dre-miR-23 is indispensable for the differentiation of endocardial cells into endocardial cushion cells in zebrafish. Moreover, dre-miR-23 inhibits TGF-*β*-induced endothelial-to-mesenchymal transition [42]. This pilot study suggests that dre-miR-23 regulates the proliferation and differentiation of cells in myocardial tissue. Nevertheless, the inhibitory effect of miR-23 may be detrimental to cardiomyocytes. rno-miR-23 facilitates cardiac ischemia/reperfusion injury by targeting glutaminase mRNA which is involved in the synthesis of glutathione [43]. We screened out that miR-23a-3p was the most statistical difference by bioinformatics analysis and experimental verification. Our study found that rno-miR-23a-3p was elevated in both intracellular and exosomal after pacing CFs. In biological function, rno-miR-23a-3p promoted ferroptosis in h9c2 cells. Knocking down miR-23a-3p has a protective effect on cardiomyocytes by increasing the expression of SLC7A11 and GPX activity, while reducing the concentration of ferrous ions and lipid peroxidation. In mechanism, miR-23a-3p mainly inhibits the translation of SLC7A11 mRNA after transcription.

The injury of oxidative stress to cardiomyocytes can be divided into contractile dysfunction and myocytes loss, while the irreversibility of myocytes loss may be pivotal in the progression of AF. Over the past decades, myriad research reported that apoptosis of atrium myocytes makes AF progress in a permanent direction. In the swine model of pacing-induced AF, Ad-siRNA-Cas-3 gene therapy reduced the expression of caspase-3 protein involved in apoptosis in atrial tissue. Moreover, electrophysiological studies have demonstrated that it also reduced the conduction heterogeneity of atrial tissue and shortened atrial conduction [44]. Clinical studies verified that when atrial tissue exhibits vast myocardial cell apoptosis or fibrosis, it affects myocardial contraction and conduction. These histological structural changes facilitate electrical remodeling, which shortens the ERP and APD, perpetuating the arrhythmia [45, 46]. Recent studies have shown that the deposition of hemosiderin in the myocardium is observed in fatal epilepsy, suggesting that ferroptosis may be a potential intrinsic mechanism leading to arrhythmia [47]. Similarly, clinical evidence using sorafenib to treat hepatic carcinoma reported a high incidence of AF in the ferroptosis inducer sorafenib group, indicating that ferroptosis would increase the incidence of AF [48]. Accordingly, as one of the end-point events of oxidative stress injury, the loss of cardiomyocytes due to ferroptosis may provide the matrix for the perpetuation of AF.

The regulation of ion channel expression by oxidative stress has been intensively studied. For instance, ROS regulates intracellular Ca^2+^ homeostasis, enhances the expression of ox-CaMKII, increases ryanodine 2-mediated Ca^2+^ release from the endoplasmic reticulum, causes the attenuation of the K^+^ currents, and shortens the APD [49]. These arrhythmogenic effects increase the susceptibility to AF. Downstream of sphingomyelinase, ceramide acts as second messenger leading to excess mitochondrial ROS [50, 51]. At the mitochondria, ceramide promotes ROS formation through increase in fission and inhibition of electron transport chain complexes [52]. In the elaborate experiments designed by Moreno et al., inhibition of sphingomyelinase and subsequent ceramide reduced hypoxia-induced vasoconstriction, whereas GW4869 decreased vasoconstriction and increased Kv1.5 in a concentration-dependent manner. Mechanistically, the neutral sphingomyelinase-derived ceramide and the activation of PKC lead to NADPH-derived ROS production, which inhibits K^+^ current and leads to vessel contraction [53–55]. It is noteworthy that GW4869 altered calcium-related ion channel expression of AF in our vivo study. But underlying mechanism of KCa3.1 and Cav1.2 remodeling should be further investigated. Our results implied that GW4869 ameliorated oxidative stress injury and the accumulation of iron. GW4869 not only reduces the output of exotic exosomes containing pernicious substances but also inhibits ROS caused by the activation of downstream signaling pathways of sphingomyelinase, thereby reducing cardiomyocytes death and delaying electrical remodeling.

In conclusion, we emphasize that first, we verified the occurrence of ferroptosis in AF and CFs promote the ferroptosis of cardiomyocytes by secreting exo-miR-23a-3p. Consequently, our results showed that the development of AF in a persistent direction can be prevented by intervening with exosomal miRNAs to reduce the loss of cardiomyocytes and oxidative stress injury.

## Figures and Tables

**Figure 1:** Human atrial tissue silico data presented exosome involved in atrial fibrillation. (a) Heat map of differentially expressed proteins. Red represents upregulated protein expression, whereas green represents downregulated protein expression. (b) Volcano plot of differential expression of mRNAs. (c) Bubble chart of GO data visualization. (d) Circular chart of enrichment analysis of involved genes and signaling pathways.

**Figure 2:** Canines electrophysiological examination by programmed stimulation and the expression of ion channel. (a) Canines electrocardiogram during programmed stimulation. In Sham group, the state at which atrial fibrillation (AF) was not reached. In Pacing group, the state at which AF was reached and the AF sustained more than 5 seconds. Compared with Pacing group, AF susceptibility attenuated by GW4869 injection because most irregular rhythm shortens than 5 seconds. (b) Effective refractory period of different parts of the atrium. GW4869 increased the ERP of RSPV and LIPV in Pacing group. (*n* =6). (c) Difference in AF inducibility, shown by the number of episodes. (*n* =6). (d) Difference in mean AF durations. (*n* =6). (e, f) Representative gel bands depicting KCa3.1 and Cav1.2 protein expression using specific antibodies. GAPDH was used as the loading control. (*n* =5). (g) Total iron level in atrial tissue. (*n* =3). (h) MDA level in atrial tissue. (*n* =3). Data are presented as the mean ± SD. Statistical significance was determined using one-way ANOVA with a post hoc Dunnett test. ∗*P* < 0.05, ∗∗*P* < 0.01, and ∗∗∗*P* < 0.001 vs. Sham group; ^#^*P* < 0.05, ^##^*P* < 0.01, and ^###^*P* < 0.001 vs. Pacing group. Abbreviations: RA: right atrium; RSPV: right superior pulmonary vein; RIPV: right inferior pulmonary vein; LA: left atrium; LSPV: left superior pulmonary vein; LIPV: left inferior pulmonary vein; dERP: dispersion effective refractory period.

**Figure 3:** GW4869 attenuates the degradation of ferroptosis-associated proteins and the secretion of exosomes in atrial tissue of rapid atrial pacing in canines. (a) Representative gel bands depicting exosome markers and ferroptosis-associated proteins expression using specific antibodies. GAPDH was used as the loading control. (b) Levels of CD63, CD81, and TSG101. (*n* =5). (c) Levels of FTH1, GPX4, and SCL7A11. (*n* =5). (d, f) Representative images of inflammatory cell infiltration, ferroptosis, fibrosis, and SLC7A11 as reflected by H&E staining, Prussian staining, Masson staining, and immunohistochemistry. (*n* =3). (e, g) Representative images of immunofluorescence staining for FTH1 protein in canines atrial tissue stimulated by rapid pacing with or without GW4869. (*n* =3). (h) RT-PCR analysis of FTH1, GPX4, and SLC7A11 expression normalized with GAPDH. (*n* =5). Data are presented as the mean ± SD. Statistical significance was determined using one-way ANOVA with a post hoc Dunnett test. ∗*P* < 0.05, ∗∗*P* < 0.01, and ∗∗∗*P* < 0.001 vs. Sham group; ^#^*P* < 0.05, ^##^*P* < 0.01, and ^###^*P* < 0.001 vs. Pacing group.

**Figure 4:** Chronological changes in ferroptosis-associated genes and oxidative stress levels in h9c2 cells after rapid pacing. (a–d) Chronological changes of FTH1, GPX4, SLC7A11, and FTL miRNAs after rapid pacing. (e, f) Representative gel bands depicting FTH1, GPX4, and SLC7A11 proteins expression in h9c2 cells stimulated by rapid pacing for 48 h and treated with or without Fer-1. (g, h) Representative gel bands depicting FTH1, GPX4, and SLC7A11 proteins expression in h9c2 cells stimulated by rapid pacing for 72 h and treated with or without Fer-1. (i, k) Representative images of immunofluorescence staining for FTH1 proteins in h9c2 cells stimulated by rapid pacing for 48 h with or without Fer-1. (j, l) Representative images of reactive oxygen species by fluoroscopy stimulated by rapid pacing for 48 h with or without Fer-1. (m, n) Mitochondrial membrane potential was detected through flow cytometry in h9c2 cells stimulated by rapid pacing for 48 h and treated with or without Fer-1. (o) Total iron level in h9c2 cells stimulated by rapid pacing for 48 h and treated with or without Fer-1. (p) MDA level in h9c2 cells stimulated by rapid pacing for 48 h and treated with or without Fer-1. (q, r) Representative gel bands depicting ion channel expression in h9c2 cells stimulated by rapid pacing for 48 h and treated with or without Fer-1. Data are presented as the mean ± SD, *n* =3. Statistical significance was determined using Student's *t* test (a–d) or one-way ANOVA with a post hoc Dunnett test (e–r). ∗*P* < 0.05, ∗∗*P* < 0.01, and ∗∗∗*P* < 0.001 vs. control group; ^#^*P* < 0.05, ^##^*P* < 0.01, and ^###^*P* < 0.001 vs. Pacing group.

**Figure 5:** Rapid pacing primary cardiac fibroblast-derived exosomes aggravate the ferroptosis of h9c2 cells. (a) Morphology of primary cardiac fibroblast-derived exosomes (CF-exos) using transmission electron microscopy. (b) Mean exosomes diameter shown by ZetaView System. (c) Exosomes were isolated from culture supernatant from CFs, dyed with phalloidin (green) and cocultured with h9c2 cells, then dyed with PKH26 (red) and viewed with fluoroscopy. (d, e) Representative gel bands depicting FTH1, GPX4, and SLC7A11 proteins expression in h9c2 cells with or without Fer-1 incubated with CF-exos for 48 h. CFs treated with or without GW4869 and stimulated by rapid pacing for 48 h and its exosomes were isolated from culture supernatant. (f) Total iron level in h9c2 cells incubated with CF-exos. (g) MDA level in h9c2 cells incubated with CF-exos. (h, i) Mitochondrial membrane potential was detected through flow cytometry in h9c2 cells incubated with CF-exos. (j, k) Reactive oxygen species was detected through flow cytometry in h9c2 cells incubated with CF-exos. Data are presented as the mean ± SD, *n* =3. Statistical significance was determined using one-way ANOVA with a post hoc Dunnett test. ∗*P* < 0.05, ∗∗*P* < 0.01, and ∗∗∗*P* < 0.001 vs. control group; ^#^*P* < 0.05, ^##^*P* < 0.01, and ^###^*P* < 0.001 vs. pacing-CF-exos group. Abbreviations: control-CF-exos: h9c2 cells incubated with control-CF-exos; pacing-CF-exos: h9c2 cells incubated with CF-exos stimulated by rapid pacing 48 h; pacing-CF-exos+Fer-1: h9c2 cells treated with Fer-1 (20 *μ*M) and incubated with CF-exos stimulated by rapid pacing 48 h; GW4869-pacing-CF-exos: h9c2 cells incubated with CF-exos treated with GW4869 (20 *μ*M) and stimulated by rapid pacing 48 h.

**Figure 6:** miR-23a-3p elevated in cardiac fibroblast-derived exosomes stimulated by rapid pacing. (a) Heat map of differentially expressed miRNAs in human atrial tissue. Red represents upregulated protein expression, whereas green represents downregulated protein expression. (b) Volcano plot of differential expression of miRNAs. (c–e) RT-PCR verification of top 8 differential expression miRNA in beagle atrial tissue, h9c2 cell, and primary cardiac fibroblast. miR-23a-3p increased significantly in beagle atrial tissue and rat cardiac fibroblasts after rapid pacing 7 days or 48 h. (f) RT-PCR analysis of miR-23a-2p expression normalized with U6 in cardiac fibroblast-derived exosomes treated with or without GW4869 (20 *μ*M) and stimulated by rapid pacing 48 h. Data are presented as the mean ± SD, *n* =3. Statistical significance was determined using one-way ANOVA with a post hoc Dunnett test. ∗*P* < 0.05, ∗∗*P* < 0.01, and ∗∗∗*P* < 0.001 vs. Sham, control, or control-CF-exos group; ^#^*P* < 0.05,  ^##^*P* < 0.01, and ^###^*P* < 0.001 vs. Pacing group or pacing-CF-exos group. Abbreviations: CF-exos, cardiac fibroblast-derived exosomes.

**Figure 7:** miR-23a-3p accelerates ferroptosis in h9c2 cells via SLC7A11 downregulation. (a) RT-PCR analysis of miR-23 in h9c2 cells transfected with miR-23a-3p inhibitor and miR-23-3p mimics, respectively. (b) RT-PCR analysis of SLC7A11 expression normalized with GAPDH after transfected with mimics and inhibitor-miR-23a-3p, respectively. (c) Total iron level in h9c2 cells transfected with mimics-miR-23a-3p. (d) MDA level in h9c2 cells transfected with mimics-miR-23a-3p. (e, f) Mitochondrial membrane potential was detected through flow cytometry in h9c2 cells transfected with mimics-miR-23a-3p and treated with or without Fer-1. (g, h) Representative gel bands depicting FTH1, GPX4, and SLC7A11 proteins expression in h9c2 cells transfected with mimics-miR-23a-3p and treated with or without Fer-1. Data are presented as the mean ± SD, *n* =3. Statistical significance was determined using one-way ANOVA with a post hoc Dunnett test. ∗, ∗∗, and ∗∗∗ indicate *P* <0.05, 0.01, and 0.001, respectively. Abbreviations: mimics: h9c2 cells transfected with mimics-miR-23a-3p (25 *μ*M) for 48 h; inhibitor: h9c2 cells transfected with inhibitor-miR-23a-3p (30 *μ*M) for 48 h.

**Figure 8:** Inhibitor-miR-23a-3p protects h9c2 cells from ferroptosis by upregulating SLC7A11. (a, b) Representative gel bands depicting FTH1, GPX4, and SLC7A11 proteins expression in h9c2 cells transfected with inhibitor-miR-23a-3p and stimulated by rapid pacing 48 h. (*n* =3). (c) Total iron level in h9c2 cells transfected with inhibitor-miR-23a-3p and stimulated by rapid pacing 48 h. (*n* =3). (d) MDA level in h9c2 cells transfected with inhibitor-miR-23a-3p and stimulated by rapid pacing 48 h. (*n* =3). (e, f) Early cell apoptosis was detected through flow cytometry in h9c2 cells transfected with inhibitor-miR-23a-3p and stimulated by rapid pacing 48 h. (*n* =3). (g, h) Representative images of reactive oxygen species by fluoroscopy in h9c2 cells transfected with inhibitor-miR-23a-3p and stimulated by rapid pacing 48 h. (*n* =3). (i) Target sequence of miR-23a-3p in the wild-type (WT) SLC7A11 3′ UTR and sequence of mutated (Mut) SLC7A11 3′ UTR predicted by starBase v2.0. (j) Measurement of firefly luciferase activity normalized to Renilla luciferase activity in 293 T cells. (*n* =5). Data are presented as the mean ± SD. Statistical significance was determined using one-way ANOVA with a post hoc Dunnett test. ∗, ∗∗, and ∗∗∗ indicate *P* <0.05, 0.01, and 0.001, respectively. Abbreviations: inhibitor: h9c2 cells transfected with inhibitor-miR-23a-3p (30 *μ*M); inhibitor+pacing: h9c2 cells transfected with inhibitor-miR-23a-3p and pacing for 48 h (30 *μ*M).

**Table 1:** Primers for qRT-PCR.

	Forward: 5′-3′	Reverse: 5′-3′	Reverse Transcription: 5′-3′
*Rat mRNA*			
FTH1	TGAGGTGTTGACTGACTTGGG	AAGCCCTGTGGCAAATCATC	
GPX4	ATACGCTGAGTGTGGTTTGC	CTTCATCCACTTCCACAGCG	
SLC7A11	ATACTCCAGAACACGGGCAG	AGTTCCACCCAGACTCGAAC	
FTL	AACCACCTGACCAACCTCCGTA	TCAGAGTGAGGCGCTCAAAGAG	
*Canine mRNA*			
FTH1	ATGTGGCTTTGAAGAACTTTGC	ATTCTCCCAATCGTCACGGT	
SLC7A11	CCCTGTATTCGGACCCATTTA	AGTTGCCTTGCTCACGTTGTT	
GPX4	AGCAATGCGGAGATCAAAGAG	GACCATACCGCTTCACCACA	
FTL	GAAACCGTCCCAAGATGAGTG	GCGGAGGTTAGTCAGGTGGT	
*miRNA*			
Let-7a-5p	CCAGCTGGGTGAGGTAGTAGGTTGT	CTGGTGTCGTGGAGTCGGCAATT	CTCAACTGGTGTCGTGGAGTCGGCAATTCAGTTGAGAACTATAC
miR-15-5p	GGGTAGCAGCACATAATGGT	CTCAACTGGTGTCGTGGAGTC	CTCAACTGGTGTCGTGGAGTCGGCAATTCAGTTGAGACAAACCA
miR-21	GTGCAGGGTCCGAGGT	GCCGCTAGCTTATCAGACTGATGT	GTCGTATCCAGTGCAGGGTCCGAGGTATTCG CACTGGATACGACTCAACA
miR-23a-3p	GCCGCGGGGTTCCTGGGGAT	GTGCAGGGTCCGAGGT	GTCGTATCCAGTGCAGGGTCCGAGGTATTCGCACTGGATACGACAAATCC
miR-27b	GGCGTGTTCACAGTGGCTAAG	CAGTGCAGGGTCCGAGGTATT	GTCGTATCCAGTGCAGGGTCCGAGGTATTCGCACTGGATACGACGCAGAA
miR-30d	GAGCTTGTAAACATCCCCGAC	AGTGCAGGGTCCGAGG	GTCGTATCCAGTGCAGGGTCCGAGGTATTCGCACTGGATACGACAGCTTC
miR-130a	GGGCTCTTTTCACATTGTGC	CTCAACTGGTGTCGTGGAGTC	CTCAACTGGTGTCGTGGAGTCGGCAATTCAGTTGAGAGTAGCAC
miR-199	GGCGTGTTCACAGTGGCTAAG	GTCGTATCCAGTGCAGGG	GTCGTATCCAGTGCAGGGTCCGAGGTATTCGCACTGGATACGACGAACAG
U6	CTCGCTTCGGCAGCACAT	AACGCTTCACGAATTTGCGT	AACGCTTCACGAATTTGCGT

## Data Availability

The data used to support the findings of this study are available from the corresponding author upon request.

## Additional Points

*Perspectives*. *Competency in Medical Knowledge*. The occurrence of ferroptosis in AF affects atrial contraction and conduction. Inhibition of the CF-exos-miR-23a-3p attenuates histological and electrical remodeling and decelerates the perpetuation of arrhythmia. *Translational Outlook*. Future studies are warranted to determine the potential therapeutic benefit of exosome inhibition and inhibitor-miR-23a-3p for the prevention of ferroptosis in AF.
